The article "Analysis of the Management Effect of Cancer Patients after Oral Chemotherapy Based on Nursing Process Reengineering" was retracted in 2023. Reasons: signs of a paper mill; suspected computer-generated content; unreliable results or conclusions; lack of ethics approval or compliance.

# Analysis of the Management Effect of Cancer Patients after Oral Chemotherapy Based on Nursing Process Reengineering

**DOI:** 10.1155/2022/4539125

**Published:** 2022-03-22

**Authors:** Yanqiong Chen, Wei Zhang, Xiang Li

**Affiliations:** ^1^Department of Radiotherapy Cancer Center, Xuzhou First People's Hospital, Xuzhoug 221116, Jiangsu, China; ^2^Oncology Department, Ningxian Second People's Hospital of Qingyang City Gansu Province, Qingyang 745200, Gansu, China; ^3^Oncology Department, Feicheng Hospital of Shandong Guoxin Yiyang Group, Feicheng 271600, Shandong, China

## Abstract

With the pollution of the environment and the acceleration of the social rhythm, the prevalence of tumors has increased year by year, and tumors have brought huge pain and inconvenience to patients. However, traditional nursing work consumes a lot of manpower and material resources, but it is difficult to improve the happiness of cancer patients, and it also brings a lot of troubles to many nursing workers. Based on the above reasons, we reengineered the traditional nursing process based on the BPR theory and applied the new process to the analysis of the management effect of cancer patients after oral chemotherapy drugs. The data shows that there are 23 patients with no pressure ulcer risk (score greater than 19) before care, 27 patients with low risk (15–19 points), 32 patients with moderate risk (13–14 points), and 18 people at high risk (less than 12 points). After nursing, there were 82 patients with no pressure ulcer risk, 10 patients with low risk, 7 patients with moderate risk, and 1 patient with high risk. This shows that the risk of pressure ulcers in patients with cancer after the use of chemotherapy drugs is significantly reduced compared with those without nursing. Nursing intervention can improve the psychological state of cancer patients during the recovery period, and nursing intervention can promote the compliance of cancer patients in various aspects of rehabilitation.

## 1. Introduction

In the clinical practice of nursing, whether the nursing process arrangement is appropriate is not only related to the patient's treatment effect, but also related to the patient's satisfaction with the medical plan [1]. Nursing process reengineering can reduce the occurrence of medical cases. It will improve nursing effectiveness and patient care satisfaction as the work goal. The development of nursing process reengineering needs to be carried out under the following conditions: the hospital management staff has paid attention to the necessity and inevitability of nursing process reengineering and can provide understanding and support; the person in charge of nursing process reengineering has a clear and clear goal of nursing process reengineering. To avoid slogan-style goals, the nursing process reengineering team has a reliable implementation effect evaluation tool [2]. Cancer patients usually have great pain. Radiotherapy, chemotherapy, or surgery and oral chemotherapy drugs will have a huge impact on the quality of life of patients and may even lead to life risks; thus, good care is especially necessary [3].

The voice based on medical care reform has always existed in academia, and there are many related studies, such as the framework of cancer patient care plan formulated by Kotenko S. The purpose of intervention is to effectively solve health problems such as insufficient self-care. Low patient compliance and decreased health quality may occur during the rehabilitation process [4]. For the first time, Mayahara *M* has carried out the continuous care model for cancer patients from the hospital to the home for the first time, a related study of nurses intervening in the early discharge of elderly patients [5]. Flanagan *J* imitates the concept of continuous care, including 6 dimensions (cross-institution, intergroup, mobility, vertical position, relationship, or individual continuity) to improve the quality of care for cancer patients [6]. Chountalas P *T* continues to improve the care model, hoping to reduce the patient's risk of chronic diseases and the quality of care [7]. Moore K proposed the concept of BPR, which uses extraction, integration, insertion, extraction, and reshaping technology to manufacture or update the initial process, creating a new process to obtain a smooth system of time, cost, quality, and service. This improvement model is in line with the current the medical environment [8]. Rega *M* L has conducted various studies on deficiencies in rational intervention, the quality of intervention strategies, intervention caregivers psychology, etc. [9]. Se established a nursing reform survey website to provide relevant information and research results on nursing reform models. After years of development, it has been widely used in the medical field in some developed countries [10].

Through the above previous studies, we can find that although many models of nursing process transformation have been proposed, many of them are based on continuity of care, and it is not enough to apply them to the analysis of the management effect of cancer patients after oral chemotherapeutics. Therefore, the main innovations of this article are as follows: (1) constructing the in-hospital tumor care process based on the BPR theory, improving the deficiencies of tumor care, saving time, and improving the rehabilitation of patients; (2) it is of practical significance to apply the modified nursing process to the management effect of oral chemotherapy drugs in tumor patients, and it will help improve the happiness of patients.

## 2. Concepts Related to the Management Effect of Cancer Patients Based on Nursing Process Reengineering

### 2.1. Concept of Nursing Process Reengineering

In clinical practice, it is found that the traditional nursing process is not flexible enough to take care of the patient comprehensively. There are many problems. The number of nurses and the function of the infirmary are still unclear. This will lead to the fact that even if nursing staff work hard, it is still difficult for patients to get high-quality care, and the quality of care for patients is impaired due to inequality in systems and capabilities [11]. Overseas, BPR has been successfully integrated into the healthcare system to restructure or improve health service processes, and this type of integrated health care application originated in the United States [12]. So far, US medical researchers have been very skilled in using BPR technology in the healthcare system. As the growing demand for health services in China, the issue of medical care arises, and BPR is used to improve processes in all aspects of hospitals, such as introducing outpatient waiting and payment, and help improve quality of service [13]. Designing new workflows specifically for nursing work can help reduce nurse mistakes, improve work quality, and increase the satisfaction of doctors and patients. Redesigning the laboratory infection control system can improve work efficiency [14]. Under the guidance of BPR theory, the process reengineering group was set up to design the process reengineering steps, principles, objectives, and other contents and reasonably and effectively evaluate the application effect of the reengineering process. The framework of nursing process reengineering based on BPR theory is shown in Figure 1.

According to the guidance of Figure 1, the working procedures of design reengineering are as follows: (1) start-up: form a process reengineering team, clarify principles, and formulate goals; (2) preliminary construction: a. original working procedure modeling; *b*. analysis, diagnosis, and redesign; (3) continuous improvement: pretest, Delphi expert consultation, and continuous improvement of the process; (4) process evaluation: process application, evaluation of the actual application effect of the process after reengineering [15]. To provide patients with more rapid and effective treatment is the common goal pursued by all relevant medical staff. Tumor care centers have been proved to be effective measures, and their standardized construction is the general trend. Currently, there is no perfect nursing process standard at home and abroad [16]. Therefore, according to the characteristics of tumor diseases and the characteristics of nursing care, it is particularly necessary to construct a more targeted, specific, operable, and widely popularized in-hospital tumor care process based on BPR theory.

### 2.2. Role and Harm of Oral Chemotherapeutics in Cancer Patients

We take irinotecan (a chemotherapeutic drug for the treatment of colorectal cancer) as an example to study the effects and risks of oral chemotherapeutics for cancer patients. With the listing of irinotecan, it has received extensive attention from researchers and doctors all over the world due to its direct efficacy [17]. In the treatment of advanced colorectal cancer, the third phase of clinical results showed that the combination of CPT-11 and 5-FU/CF was significantly higher than 5-FU/CF in terms of survival and remission. Irinotecan has also become the European Union and the first chemical drug used by the US FDA to treat advanced colon cancer [18]. CPT-11 and oxaliplatin combined with leucovorin and 5-FU light have a better effect in the treatment of patients with gastrointestinal cancer. Folinic acid can stabilize the synthesis of 5-FU and thymidine synthase and increase 5-FU with parathymidine Inhibition of chemical synthase [19]. Studies have shown that the first chemotherapeutic drug CPT-11 is also slowly being used to treat gliomas. It can be used in combination with cisplatin to treat small cell lung cancer and has obvious clinical effects. The combination of CPT-11 and gemcitabine is well tolerated and has less toxicity in the treatment of pancreatic cancer. In addition, CPT-11 is also used to treat esophageal cancer, cervical cancer, leukemia, etc. The toxic and side effects during treatment are mainly intestinal reactions, adverse reactions of the blood system, and complex symptoms such as hair loss, fatigue, mucositis, and skin toxicity (including hand-foot syndrome) [20]. Existing studies believe that, from the perspective of drug metabolism, this is mainly due to the toxicity of the central metabolite of CPT-11. The occurrence of diarrhea may be due to the direct damage of SN-38 to the intestinal tract [21]. Intestinal flora, such as *Escherichia coli*, *Clostridium perfringens*, and *β*-glucuronidase produced by Bacteroides, can convert SN-38G back to SN-38, thereby destroying the intestinal epithelium and reducing intestinal inflammation. The contact time of SN-38 with the intestinal epithelium and the concentration in the intestine are the key to causing delayed diarrhea [22]. Therefore, it is necessary to care for tumor patients with oral chemotherapy drugs. Good care can effectively reduce the serious adverse reactions caused by chemotherapy drugs.

### 2.3. Hospital Nursing Business Process Reengineering Based on Deep Learning

Deep learning technology originated in neuroscience. Since current deep neural networks mainly use convolutional structures, deep neural networks are sometimes called deep convolutional neural networks [23]. After the rise of deep neural networks, researchers have found that letting neural networks automatically learn is very effective. The method of automatically learning features is usually called “representational learning” by researchers. The deep learning model has a very powerful feature extraction ability, which avoids the inefficiency and cumbersomeness of manually designing features. Since deep learning features are automatically learned, deep learning is feasible for the application of hospital care business process reengineering. Therefore, the use of neuron shared weights greatly reduces the number of parameters that need to be trained in the neural network [24]. In addition, the shared weight strategy used can be used to convolve the image data to achieve the forward propagation of the neural network (the filter is composed of weights). A convolutional neural network usually includes a convolutional layer, a pooling layer, a fully connected layer, and a loss layer (needed in the training phase, not required in the testing and deployment phases). A binary classification network with 2 convolutional layers, 2 pooling layers, and two fully linked layers (the last fully-linked layer is used for classification) is shown in Figure 2.

In the fully linked layer of the neural network, when calculating the output of a layer, the weight vector used by each neuron of the output is different.  Figure 3 is the two-class convolutional neural network.

As shown in Figure 3, the *L* layer has 2 neurons, the L-1 layer has 4 neurons, and the weight matrix of the *L* layer is 2^*∗*^4. The two neurons in the *L* layer use different weight vectors; that is, the row vectors of the nonshared matrix on the right are used, respectively [25]. The weighted input and output calculation formulas of the *L* layer are shown in (1) and (2), where *z* represents the weighted input of the jth neuron of the *L* layer, *a* represents the output of the jth neuron of the *L* layer, and *b* represents the jth neuron of the *L* layer. The bias of each neuron *x* represents the activation function, and *w* represents the connection weight from the nth neuron in the *L*−1 layer to the jth neuron in the *L* layer:

(1) $$\begin{array}{c} \text{z}=\sum_{k=0}wa\left(L-1\right)+b,j=0,1, \end{array}$$

(2) $$\begin{array}{c} a=x\left(z\right),j=0,1. \end{array}$$

When performing convolution operation in image processing, the convolution kernel needs to be flipped 180° first [26, 27]. The two-dimensional discrete convolution operation formula in image processing is shown as follows:

(3) $$\begin{array}{c} M\left(x,y\right)=\left(W*I\right)\left(x,y\right)=\sum \sum W\left(s,t\right)I\left(x-s,y-t\right), \end{array}$$

in which *I* represents the input image, *W* represents the convolution function, and *M* represents the output of the convolution operation. Unlike image processing, the so-called “convolution” in deep neural networks is a correlation function, or cross-correlation function, as shown in the following equation:

(4) $$\begin{array}{c} M\left(x,y\right)=\left(W*I\right)\left(x,y\right)=\sum \sum W\left(s,t\right)I\left(x+s,y+t\right). \end{array}$$

This formula is almost the same as the convolution operation (3), but the core W is not flipped. In the neural network, although the realization is related operations, in the deep neural network, the size of the neurons in the *L* layer is 2^*∗*^2, the size of the neurons in the L-1 layer is 4^*∗*^4, and the size of the shared weight matrix of each neuron in the *l* layer is 3^*∗*^3. The weighted input and output calculation formulas of the *l* layer can be expressed by (5) and (6):

(5) $$\begin{array}{c} \text{z}=\sum_{i=0}\sum_{l=0}wa\left(l-1\right)+b, \end{array}$$

(6) $$\begin{array}{c} \text{al}=x\text{z}\left(x,y\right)=0,1. \end{array}$$

Among them, *z* represents the weighted input of the *l* layer of neurons, al represents the output of the *l* layer of neurons, *b* represents the shared bias of the *l* layer of neurons, and *x* represents the activation function. Common activation functions are sigmoid function, Tanh function, and ReLu function, and they are as follows:

(7) $$\begin{array}{c} xz\left(x,y\right)=\frac{1}{1+e^{\left(-z\left(x,y\right)\right)}},\\ xz\left(x,y\right)=\frac{e^{z\left(x,y\right)}-e^{-z\left(x,y\right)}}{e^{z\left(x,y\right)}+e^{\left(-z\left(x,y\right)\right)}},\\ x\text{z}\left(x,y\right)=\text{max}\left(0,z\left(x,y\right)\right). \end{array}$$

Suppose that the Softmax classification is performed in the *L* layer of the neural network (the last layer is fully linked) [28]. The *L* layer has a total of *n* neurons. The weighted input and output calculation formulas of the *L* layer are shown in (8) and (9):

(8) $$\begin{array}{c} \text{z}=\sum_{n}wa_{n}+b_{j}, \end{array}$$

(9) $$\begin{array}{c} a=\frac{e}{\sum {}_{n}e^{z}}, \end{array}$$

in which *z* represents the weighted input of the *L* layer neuron, and *a* represents the output of the *L*-1 layer neuron [29–31]. *a* can be understood as the probability of classifying the sample. It can be seen from (9) that the sum of the outputs of all neurons in the *L* layer is equal to 1.

(10) $$\begin{array}{c} \sum_{j=1}^{n}a_{j}^{L}=1. \end{array}$$

The softmax loss function formula is shown in (13).

(11) $$\begin{array}{c} Z=-\frac{1}{\text{n}}\left[\sum_{i=1}\sum_{j=1}^{n}1\left(y=j\right)\log\;a^{L}\right]. \end{array}$$

This formula is the loss function of *n* samples, and *y* represents the label of the *i*th sample. The value range of 1(*y* = *j*) is only 0 and 1. When the bracket equality holds, it takes 1, and it takes 0 if it does not. It can be seen from (11) that the loss function formula of a single sample *x* is shown in (14).

(12) $$\begin{array}{c} C=-\log\;a_{y}^{L}. \end{array}$$

Suppose that the loss function requiring optimisation is C (o1, o2, ... , on), assign the *o* an initial value, and then let it change a small increment, so that the target function also produces a small change, constantly iterating the process. When the loss function is C almost no longer changes, it is assumed that the function has reached the optimal value. It is known from calculus knowledge that when the *v* changes a small increment, the increment of the loss function C can be expressed by its full differential, as shown in (15).

(13) $$\begin{array}{c} \nabla C\approx \frac{\partial C}{\partial {\text{o}}_{1}}\nabla v_{1}+\frac{\partial C}{\partial {\text{o}}_{2}}\nabla v_{2}+...+\frac{\partial C}{\partial {\text{o}}_{\text{n}}}\nabla v_{n}. \end{array}$$

▽C can be written as follows:

(14) $$\begin{array}{c} \nabla C\approx C*\nabla \text{v,} \end{array}$$

in which C and ∆v are shown in (15) and (16):

(15) $$\begin{array}{c} C=\left(\frac{\partial C}{\partial {\text{v}}_{1}},\frac{\partial C}{\partial {\text{v}}_{2}},...,\frac{\partial C}{\partial {\text{v}}_{n}}\right), \end{array}$$

(16) $$\begin{array}{c} \nabla \text{v}={\left(\nabla {\text{v}}_{1},\nabla {\text{v}}_{2},...,\nabla {\text{v}}_{\text{n}}\right)}^{\text{T}}. \end{array}$$

Assume that ∆v is shown in

(17) $$\begin{array}{c} \nabla \text{v}=-\zeta \nabla C. \end{array}$$

However,

(18) $$\begin{array}{c} \nabla \text{C}=-\zeta {\left\|\nabla C\right\|}^{2}, \end{array}$$

in which ▽*C* ≥ 0 guarantees *C* ≤ 0. That is, if *v* changes according to the rule in (17), then the loss function C will always decrease and will not increase. After constructing a deep neural network, the next task is to train the network. To train a neural network using the gradient descent method, firstly initialize the weights, and the quality of the initialization method will affect the convergence speed of the neural network.

## 3. Experimental Analysis of the Management Effect of Nursing Process Reengineering on Cancer Patients after Oral Administration of Chemotherapeutics

### 3.1. Reengineering the Nursing Process in the Hospital Based on BPR Theory

Nursing process reengineering should first determine the principles of nursing process reengineering: (1) patient-centered; (2) safety-based; (3) fast and efficient process operation as the goal; (4) continuous improvement as the concept. Formulate process reengineering goals: (1) after reengineering, the process has strong operability, which can ensure smooth progress of nursing intervention, high efficiency of rescue work, and reduction of patient tumor delay time; (2) through process reengineering, clarify the scope of work of nurses in the nursing process, and improve the coordination of medical and nursing care; (3) after the reengineering process, a clear time system and responsibility system are established to reduce the dependence of nursing work on the experience of tumor nurses; (4) the reengineered process needs to run on the basis of the original process and be stable and smooth and does not conflict with the existing overall system or other single department systems. Currently, there is basis for nursing process standards, and nurses in various hospitals also carry out nursing work based on their own experience, and the work content is similar. We take the tumor care work content of a hospital as a prototype and model the original care process as shown in Figure 4.

As shown in Figure 4, after the original nursing process of the hospital is determined, interviews with the medical staff of the hospital are conducted to understand their understanding of the current nursing situation in the hospital and their suggestions for improvement. The interviewees are first-line nurses with more than 5 years of work experience in the emergency department. During the interview, data collection and analysis are carried out at the same time, and all the relevant work of one respondent is completed before the interview with the next respondent occurs. After repetition of the theme of the materials, the semistructured interview was deemed to be saturated with information, and the interview was ended. In the end, this study interviewed 8 interviewees, all of whom were emergency department nursing team leaders. The specific conditions are shown in Table 1.

Through comprehensive analysis and extraction of all interview data, and analysis and summary of interview results, the following questions are obtained: 1. patients' treatment process is unreasonable, which greatly increases the ineffective workload of doctors; 2. the hospital has not notified the patients immediately upon admission, and the definition of the time of admission is unclear; 3. improper use of the green channel; 4. there are conflicts in hospital time management. Some of the accompanying doctors in the transfer of patients are not the doctors in charge of the patients, and they do not know enough about the patients' conditions to obtain complete information; 5. unreasonable assignment of tasks, etc. According to the above conclusions, the nursing process in the hospital was continuously improved. Meanwhile, the preliminary experiment was conducted for comparative analysis. The results are shown in Table 2.

It can be seen from Table 2 that the time of *D* to ECG was shortened (*P* < 0.05), and the time of *D* to TnI was shortened (*P* < 0.05) of patients in the pretest group. It is proved that the implementation of the nursing process in the hospital is related to the shorter diagnosis time of the patient. However, there was no significant difference in the emergency stay time and *D* to B time of the two groups of patients. The pretest not only verified the effect of the process implementation, but also constantly discovered the problems in the practice of nursing process transformation during the pretest and further modified it to ensure the actual operability of the process. The results of the expert's inquiry on the process structure evaluation form after the nursing process transformation are shown in Table 3.

As can be seen from Table 3, experts agree on item 7 but disagree on items 3, 4, and 5. However, the analysis found that the experts with different opinions have professional or regional characteristics. For example, the main content of item 3 is the content of patient evaluation. The two experts with different opinions are all cardiologists, which may be caused by insufficient understanding of the working conditions of the triage nurse. However, entries 4 and 5 are most likely to be caused by unit characteristics. The experts with different opinions in the two entries come from the special specialized heart hospitals, so they may lead to inconsistent with the evaluation level of experts in other general hospitals. Finally, for items 3, 4, and 5, they chose to adopt the opinions of most experts. For individual experts with different opinions, once again communicating with the experts and further explaining the reasons for not adopting them, the experts said that they could understand and agree.

### 3.2. Evaluation of the Rehabilitation Effect of Patients after Nursing Process Reengineering

A presurvey was conducted between 2020 and 2021 using the method of randomization. 100 cancer patients who met the inclusion criteria in a certain hospital were selected and divided into two groups. The intervention group used the reengineered care method, and the control group used the original care method. During the hospitalization period, patients will be given routine care measures, and health education about diseases will be explained to patients in words that are easy for the patient to understand, including knowledge about the oral chemotherapeutics and tumor, reasonable diet, and early exercise. Comparison of demographic variables between the two groups of patients is shown in Table 4.

It can be seen from Table 4 that the experimental subjects are between 45 and 80 years old, the evaluation age is 57.82 ± 12.31, the average age of the intervention group is 58.14 ± 12.31, the average age of the control group is 57.01 ± 6.32, and the *P* value of the two 0.811 is greater than 0.05, and there is no statistical difference between the two. The gender of the two groups was also not statistically significant, but there were more males than females in the study, and there was no statistical difference in the marital status of the two groups of patients, and more than 90% of the study subjects were married. The comparison of BI index values between the two groups of patients before and after intervention is shown in Figure 5.

It can be seen from Figure 5 that the BI index value distribution of the two groups of patients before and after the intervention is in accordance with the normal distribution, and the variance is homogeneous. The BI index of the two groups of patients was compared using the two independent sample *t*-test method in statistics. After comparing the BI index of the two groups of tumor patients before transformation, *P*=0.805, there is no statistical difference. After the transformation, the BI index value of the two groups was compared *P*=0.006, and the results were statistically different. The results of the intervention can show that the nursing transformation intervention can improve the patient's daily activity ability. The comparison of the anxiety and depression scores of the two groups of patients before and after intervention is shown in Figure 6.

It was tested that the distribution of anxiety scores of the two groups of patients before and after the intervention accorded with the normal distribution, and the variance was homogeneous, and the anxiety scores after the intervention showed homogeneous variance after the square root transformation. The anxiety scores of the two groups of cancer patients before intervention were compared, and the results showed that the *P* values were all greater than 0.05, and there was no statistically comparable difference. After 3 months of intervention, the *P* values of the anxiety and depression scores of the two groups of patients were all less than 0.05, and the results were statistically different, reflecting the positive effect of continuous nursing intervention on the psychological state of cancer patients. The rehabilitation compliance comparison of the two groups of patients after intervention is shown in Figure 7.

It can be seen from Figure 7 that, after the use of chemotherapy drugs, the two groups of cancer patients have little difference in compliance with the balanced diet and rational drug use. The balanced diet intervention group complied with 37 people, partially complied with 9 people, and did not comply with 5 people, the control group. In the intervention group, 33 people complied well, 9 people partly complied, and 10 people did not comply. There were 21 people in the reasonable medication intervention group with good compliance, 29 people in the control group, 11 people in the partially compliant intervention group, 12 people in the control group, 18 people in the noncompliant intervention group, and 10 people in the control group. After comparing the compliance of these two items, the *P* value is greater than 0.05, which is not statistically significant. There are large differences in compliance with the five items of smoking cessation, alcohol restriction, exercise time, exercise frequency, physical activity, and self-test. The results are statistically different, and the effect of physical activity is the most significant, with the largest difference. There were 23 people in the control group with good physical compliance, 38 people in the intervention group, 10 people in the partial compliance control group, and 8 people in the intervention group.

### 3.3. Analysis of the Management Effect of Cancer Patients after Oral Chemotherapy Based on Nursing Process Reengineering

Oral chemotherapy is one of the most important treatments for patients with malignant tumors, but oral chemotherapy can cause many adverse reactions, such as nausea, vomiting, and anorexia. Nausea and vomiting after oral chemotherapy (CINV) not only affect the quality of life of cancer patients, but also severely reduce the patient's compliance with treatment, which makes the patient resistant to further chemotherapy, leading to the suspension of effective treatment. Therefore, nursing care is necessary for patients with oral chemotherapy drugs. At the same time, the level of care for patients with different living abilities should be different. The comparison table for the self-care ability of patients is shown in Table 5.

It can be seen from Table 5 that there are 56 self-care patients who take medication, 124 are partly dependent, 31 are unable to take care of themselves at all, 20 of the patients without medication can take care of themselves, 158 of them need to be partially dependent on their lives, and some are completely unable to take care of themselves. Of the 24 patients, 31 of the surgical patients were able to take care of themselves, 142 were partially dependent, and 26 were unable to take care of themselves at all. According to McNemar-Bowker test, the difference in self-care ability of patients before and after surgery is statistically significant. The patient's pressure ulcer risk assessment is shown in Figure 8.

It can be seen from Figure 8 that patients with chemotherapy drugs had 23 without pressure sores (score greater than 19), 27 with low risk (15–19), 32 with moderate risk (13–14), and 18 with high risk (below 12). After nursing, there were 82 patients with no pressure ulcer risk, 10 patients with low risk, 7 patients with moderate risk, and 1 patient with high risk. Pressure ulcers occur because the patient's long-term bed rest and turning over reduce pressure on the tissues, causing nutritional imbalance and circulatory disorders in the compressed parts, and progressively worsening, eventually leading to soft tissue necrosis. It is one of the three major complications of clinical care. If a pressure ulcer occurs, it will not only have a negative impact on the patient's treatment effect, but also reduce the patient's quality of life, which can even endanger the patient's life in severe cases. However, through this study, it can be seen that the risk of pressure ulcers after the use of chemotherapeutic drugs is significantly reduced, and the risk of pressure ulcers in patients without medication is higher than that of pressure ulcers with medication. A fall is a sudden, nonsubjective change in body position and falling to the ground or lower planes. Inpatients have different risks of falling due to age, severity of illness, familiarity with the environment, and change of caregivers. There are reports showing that the incidence of falls in hospitalized patients is 3 to 7 per thousand, but it has become an important safety issue affecting the health of patients. The risk assessment of the patient falling from the bed is shown in Figure 9.

It can be seen from Figure 9 that, among the patients taking chemotherapy drugs, 34 were at high risk of falling from bed (>12 points) before care, and 32 were at risk of falling from bed (8–12 points), and there was no risk of falling from bed (<8 points); there are 34 people. After nursing, the number of patients without the risk of falling from bed increased to 73, the number of patients with risk of falling from bed was 12, and only 15 patients were at high risk. Among the patients without medication, 26 were not at risk of falling and falling before nursing, 47 were at risk, and 27 were at high risk. After nursing care, the number of people who were not at risk of falling from bed rose to 63, 20 were at risk, and only 17 were at high risk. It can be seen that the difference in fall risk assessment after nursing is statistically significant. Once a fall occurs, patients are prone to coexisting diseases or injuries, length of stay in hospital, and medical expenditures increase. Preventing falls is an important part of nursing work, and it is also an important index to evaluate the safety and nursing quality of hospital patients. Tumor patients are prone to limb discomfort due to the lesion invading normal brain function areas, which is one of the high-risk factors for falling and falling from the bed. The damage to the patient's brain tissue and the resulting impaired consciousness caused by the medication can cause the patient to develop postoperatively, the main reason for the fall. The use of special drugs after medication is also a risk factor for falls. The mobility of cancer patients has also changed after medication. The proportion of patients who can move on their own after taking the medicine is greatly reduced, as shown in Figure 10.

It can be seen from Figure 10 that 11 of the cancer patients treated with chemotherapy drugs were able to move normally before nursing, which increased to 36 after nursing, 43 were active at the bedside before nursing, and 24 were active in bed after nursing. There were 26 patients before, and it was reduced to 28 after care. There were 20 patients before care for bedridden patient, and only 12 after care. For untreated patients, before nursing, 18 were normal patients, 23 were bedside active patients, 34 were only able to move in bed, 25 were bedridden patients, and 31 were able to move normally after care. 46 people can move around the bed, 12 people move on the bed, and 11 people sleep on the bed. It can be seen that the patient's mobility is greatly improved after nursing, the number of bedridden patients is reduced, and the patient's mobility after chemotherapeutic drugs is relatively improved compared to unused patients, but it is not obvious.

## 4. Discussion

Nursing process reengineering refers to the adjustment and improvement of nursing work process by studying and analyzing the problems exposed in the previous nursing work and the reasons leading to the problems, so as to reduce medical and nursing accidents and improve the effectiveness of nursing and patients' nursing satisfaction as the work goal. In the process of nursing process reengineering, patients' service needs should be taken as the core, not exceeding the requirements of relevant norms and systems, and efforts should be made to innovate the service process. Tumor brings great pain and life pressure to people. The usual chemotherapy and surgical treatment usually cost high, and the postoperative damage to the human body is large, so oral chemotherapy is gradually becoming a common treatment, but the side effects of chemotherapy are relatively large, and patients need good nursing conditions. By comparing the management effect of hospital nursing process reengineering on tumor patients after oral chemotherapy, we found the following.

The research is based on mature and applicable BPR theory and has scientific and systematic reengineering steps. By shortening DtoECG time and DtoTnI time, the established AMI emergency nursing process can accelerate the diagnosis of patients. The hospital AMI emergency nursing process established by the institute adopted a clear responsibility system, which solved the problems mentioned in the interview, such as repetitive work among nurses and difficulties for junior nurses to cope with. Nurses are also trained to improve their comprehensive ability, enhance their self-motivation in the process of work, improve their EXPERIENCE of AMI rescue, and enhance the sense of belonging of nurses.

Although our country pays more and more attention to nursing, there are still more problems in the nursing process. Through the reform of the nursing process, we can find that the daily activities of the two groups of patients have improved after nursing. It is because this ability can be improved through self-training and self-adaptation. The results of anxiety and depression symptoms of patients before and after nursing were statistically different, and the patients' anxiety symptoms decreased significantly. The reason may be that as the patient's condition gradually relieved, the anxiety symptoms decreased. The results of the compliance comparison before and after patient care showed that there were statistical differences in the compliance of the five items of smoking cessation, alcohol restriction, exercise time, exercise frequency, physical activity, and self-test. There was no statistical difference in the compliance of the two items of medication.

The Barthel index scoring method was used to evaluate the self-care ability of patients, individualized care was given to patients according to different grades, and attention was paid to mobilize the self-care potential and enthusiasm of patients, guiding patients to actively participate in nursing and self-care. Because of the difference of nursing score, the nursing patients in the daily living ability have been significantly improved, so the basic care and specialized care of tumor patients are also particularly important. In addition to the implementation of comprehensive basic nursing, but also taking the initiative to analyze potential dangers, do a good job of safety precautions, timely eliminate risk factors, prevent accidents, and ensure the personal safety of patients, so as to improve the quality of nursing. In this study, by comparing the two groups of tumor patients, it was found that the low risk and high risk scores of tumor patients were significantly higher than before nursing, indicating that the risk index of pressure ulcers rose before and after nursing. How to effectively prevent pressure ulcers is the focus of cancer patients nursing.

## 5. Conclusions

Nursing process reengineering improves the professional knowledge level of nurses. Nursing process reengineering requires the establishment of a nursing management team. The management team conducts investigations, analyzes and solves the problems in traditional nursing, formulates new nursing process plans, and makes modifications after preliminary trials. For the management effect of cancer patients after oral chemotherapy, we can find that the pretest not only verifies the effect of the process implementation, but also constantly discovers the problems in the practice of the nursing process transformation during the pretest process and further modifies it to ensure the actual process. The modified nursing intervention effect is better than the conventional hospital nursing effect. The modified intervention can improve the ability of daily life of cancer patients during the rehabilitation period. Nursing intervention can improve the psychological state of cancer patients during the rehabilitation period. Nursing intervention can promote the various aspects of cancer patients, rehabilitation compliance. After using chemotherapy drugs, the risk of pressure ulcers after the patients are treated is significantly reduced. The risk of pressure ulcers in patients without medication is higher than the risk of pressure ulcers with medication, and the risk of patients falling from bed can be effectively reduced.

## Figures and Tables

**Figure 1:** The framework of nursing process reengineering based on BPR theory.

**Figure 2:** Two-class convolutional neural network.

**Figure 3:** Two-class convolutional neural network.

**Figure 4:** The original care flowchart after modeling.

**Figure 5:** Comparison of BI index values between the two groups of patients before and after intervention.

**Figure 6:** Comparison of anxiety scores between the two groups of patients before and after intervention.

**Figure 7:** Comparison of rehabilitation compliance between the two groups of patients after intervention. (a) Intervention group. (b) Control group.

**Figure 8:** The patient's pressure ulcer risk assessment chart. (a) Medication. (b) No medication.

**Figure 9:** Comparison of the evaluation scores of tumor patients before and after medication. (a) Medication. (b) No medication.

**Figure 10:** Activity of cancer patients before and after care. (a) Medication. (b) No medication.

**Table 1:** General information of interviewees.

Gender	Age	Production	Blood flow	Working years
Female	30	Head nurse	Undergraduate	6
Female	31	Head nurse	Postgraduate	5
Female	33	Head nurse	Undergraduate	8
Male	32	Head nurse	Junior college	8
Female	40	Deputy chief nurse	Postgraduate	11
Female	28	Head nurse	Undergraduate	5
Female	34	Head nurse	Undergraduate	7
Female	33	Head nurse	Junior college	9

**Table 2:** Comparison of time nodes between the control group and the pretest group.

Outcome indicators	Control group	Preexperimental group	*T*/*Z*	*P* value
D to ECG	3.27 ± 2.266	1.86 ± 0.823	*T* = 2.163	0.031
D to TnI	20.31 ± 3.821	17.63 ± 3.612	*T* = 3.265	0.004
Emergency stay	40.12 ± 21.03	26.13 ± 19.65	*Z* = 0.168	0.831
D to B	65.12 ± 23.21	70.23 ± 22.13	*Z* = 0.367	0.613

**Table 3:** Delphi supplementary content evaluation form letter inquiry results.

Entry	Main content	Yes		No	
		Frequency	Percentage	Frequency	Percentage
1	Triage time	16	100	0	0
2	Precedence	13	93	2	6.6
3	Evaluation content	13	93	2	6.6
4	Vital signs measurement	12	86	3	12.3
5	Electrocardiogram	13	93	1	3.3
6	Experience requirement	16	100	0	0
7	Assessment requirements	16	100	0	0

**Table 4:** Demographic variables of the two groups of patients.

Variable		Research object	Intervention group	Control group	*P* value
Age		57.82 ± 12.31	58.14 ± 12.31	57.01 ± 6.32	0.811
Gender	Male	56	30	26	0.920
	Female	44	21	23	

Marital status	Married	96	46	50	0.779
	Unmarried	4	3	1	

**Table 5:** Comparison of self-care ability of patients with glioma before and after surgery.

	Take care of yourself	Partial dependence	Totally dependent on	*P* value
Medication	56	124	31	<0.001
No medication	20	158	24	
Operation	31	142	26	

## Data Availability

The simulation experiment data used to support the findings of this study are available from the corresponding author upon request.
